# Effect of Transcatheter Arterial Chemoembolization Combined with Radiofrequency Ablation on Liver Function and Immune Function in Patients with Hepatocellular Carcinoma

This article has been retracted.

**DOI:** 10.1155/2022/4842370

**Published:** 2022-09-27

**Authors:** Yan Zhou, Ying Qian, Weiming Xiong, Naijun Yan, Bing Hu, Zhiyuan Xiong, Weixin He

**Affiliations:** ^1^Department of Liver Disease and Infection, 906 Hospital of PLA, Ningbo 315040, Zhejiang, China; ^2^The First College of Clinical Medical Science, Three Gorges University & Yichang Central People's Hospital,Yichang, Hubei 443008, China

## Abstract

**Objectives:**

To investigate the effects of transcatheter arterial chemoembolization (TACE) combined with radiofrequency ablation (RFA) on liver function and immune function in patients with hepatocellular carcinoma (HCC).

**Methods:**

From December 2016 to January 2019, patients with primary liver cancer who could not be operated on were selected as the study subjects. 170 patients were randomly divided into two groups. The control group was treated with transcatheter arterial chemoembolization (*n* = 85). The patients in the observation group were treated with transcatheter arterial chemoembolization combined with radiofrequency ablation (*n* = 85). The clinical effects of the two groups were analyzed. The changes of liver function and immune function were detected by automatic biochemical analyzer before and after treatment. The changes of hypoxia inducible factor-1 (HIF1) alpha and vascular endothelial growth factor (VEGF) levels before and after treatment were analyzed by enzyme-linked immunosorbent assay (ELISA).

**Results:**

The total effective rate in the observation group was significantly higher than that in the control group (*P* < 0.05). After treatment, serum levels of alanine aminotransferase (ALT), aspartate aminotransferase (AST), CD8+, HIF1 alpha, and VEGF decreased significantly (*P* < 0.05), while levels of total bilirubin, direct bilirubin, indirect bilirubin, CD3+, CD4+, and CD4+/CD8+ increased significantly (*P* < 0.05). The changes of the above indexes in the observation group were more significant than those in the control group (*P* < 0.05).

**Conclusion:**

Hepatic arterial chemoembolization combined with radiofrequency ablation has a significant effect on liver function and immune function in patients with liver cancer, which may be related to the abnormal levels of HIF1*α* and vascular endothelial growth factor.

## 1. Introduction

Primary liver cancer is one of the common malignant tumors in our country. The etiology and pathogenesis of primary liver cancer have not yet been determined. At present, it is believed to be related to gene mutation and soil and water factors [1]. The main symptoms are liver pain, fatigue, weight loss, abdominal distension, loss of appetite, etc., which will harm surrounding organs and cause rupture and bleeding. Early surgical resection is the most effective treatment method, and postoperative comprehensive treatment can be based on the patient's condition and combined with drugs. The prognosis of primary liver cancer is closely related to early diagnosis and early treatment [2, 3].

Hepatic arterial chemoembolization is currently the first choice for the clinical treatment of advanced hepatocellular carcinoma, which has obvious effects on inhibiting tumor vascular invasion and relieving tumor progression [4]. Radiofrequency ablation is a minimally invasive interventional surgery for the clinical treatment of solid tumors, which belongs to the category of thermal ablation [3]. The rapid proliferation of tumor cells is usually accompanied by hypoxia in the organized microenvironment, and VEGF and HIF1*α* are important participants in this physiological process [5]. This study analyzed the effect of hepatic arterial chemoembolization combined with radiofrequency ablation on liver function and immune function in patients with liver cancer, in order to provide reference for clinical treatment.

## 2. Materials and Methods

### 2.1. Research Objects

The subjects were patients with inoperable primary liver cancer who were admitted to our hospital from December 2016 to January 2019. Inclusion criteria were as follows: all study subjects were pathologically confirmed to be with primary liver cancer and could not continue surgery, liver function Child grade was A or B, age ≥45 years, complete clinical data, normal mental state, consent to this study, and compliance with the requirements of the hospital ethics committee. Exclusion criteria were as follows: patients with other malignant tumors, patients with severe metabolic system diseases, patients with organic heart or kidney disease or severe dysfunction, patients with incomplete clinical data, mental illness and uncooperative patients, and patients with contrast medium allergy. 170 patients were divided into two groups by the random data table method: control group patients received hepatic arterial chemoembolization, and observation group received hepatic arterial chemoembolization combined with radiofrequency ablation. In the control group, there were 44 males and 41 females, aged 45–67 years (56.6 ± 11.3), 52 patients with Child liver function grade A, and 33 patients with B. In the observation group, there were 43 males and 42 females, aged 45–65 years (56.2 ± 11.8). There were 50 patients with Child liver function grade A and 35 patients with B. There was no statistical difference between the two groups in general data such as sex ratio, average age, and Child–Pugh classification [6] of liver function (*P* > 0.05).

### 2.2. Methods

Patients in the control group received hepatic arterial chemoembolization: the modified Seldinger method was used to perform femoral artery puncture, catheters were inserted into the common hepatic artery, left and right hepatic arteries, and proper hepatic artery, and arteriography was performed. Chemotherapy drugs (oxaliplatin J20150117) and embolic agents (liquid lipiodol) are injected. The corresponding lipiodol and pirarubicin suspension were selected according to the size of the liver cancer lesions of the research subjects. At the same time, gelatin sponge particles were used for thromboembolism according to the actual situation. Hepatic arterial chemoembolization was performed at an interval of 2 months, and relevant indicators were observed after 3 treatments. The observation group was treated with hepatic arterial chemoembolization combined with radiofrequency ablation. The control group underwent radiofrequency ablation after 4 weeks of hepatic arterial chemoembolization, which was the same as the observation group. Under the precise guidance of CT, radiofrequency ablation was performed after puncture at the appropriate location. Participation in radiofrequency ablation therapy was adjusted according to the size, location, and morphology of the patient's tumor. The treatment principle from far to near is adopted from the epidermis, and the ablation method of multiple overlapping and multiple needle overlapping is used for treatment.

### 2.3. Observation Indicators and Analysis Methods

The clinical treatment effect includes medium [7]: complete remission (CR) refers to the disappearance of the target lesion after the patient receives treatment, and it is maintained for at least four weeks; partial remission (PR) is a 30% reduction in the sum of the maximum diameters of the patient's baseline lesions after treatment, maintained for at least four weeks; stable (SD) is the reduction in the sum of the maximum diameters of the baseline lesions but less than 30% after the patient receives treatment; progressive (PD) refers to patients whose baseline lesions did not decrease or even increase after treatment. Total effective rate = (CR cases + PR cases + SD cases)/total cases × 100%.

The changes of liver function and immune function in the two groups of patients before and after treatment were detected. CD3/CD4/CD8 detection kits were purchased from Shenzhen Ruijing Biotechnology Co. Ltd. ALT and AST detection kits were purchased from Nanjing Jiancheng Bioengineering Institute; total bilirubin, direct bilirubin, and indirect bilirubin detection reagents were purchased from Roche. The automatic biochemical analyzer is Roche Cobas8000c701. The changes of HIF1*α* and VEGF levels before and after treatment were analyzed by enzyme-linked immunosorbent assay. HIF1*α* detection kit was purchased from R&D Company; VEGF detection kit was purchased from CST Company. The full-wavelength microplate reader is RT-6100 of Redu Company.

### 2.4. Statistical Analysis Data

Statistical analysis was done by SPSS18.0 statistical software, the count data were expressed as percentage, and the comparison between two groups was done by x2 test; measurement data were expressed as mean ± standard deviation, *t*-test was used for comparison between two groups, and paired *t*-test was used for comparison within group before and after treatment. *P* < 0.05 means the difference is statistically significant.

## 3. Results

### 3.1. Comparison and Analysis of the Clinical Effective Rate of the Two Groups of Patients

The study found that the total effective rate of patients in the observation group was significantly higher than that of the patients in the control group, and the difference was significant (*x*^2^ = 2.449, *P* < 0.05), as shown in Table 1.

### 3.2. Changes of Liver Function Index Levels before and after Treatment in the Two Groups of Patients

The study found that the levels of serum transaminases ALT and AST in the two groups of patients after treatment were significantly decreased (*P* < 0.05), while the levels of total bilirubin, direct bilirubin, and indirect bilirubin were significantly increased (*P* < 0.05), and the changes of the above indicators in the observation group were more obvious than those in the control group (*P* < 0.05), as shown in Tables 2 and 3.

### 3.3. Comparison of Changes in Immune Function Indexes between the Two Groups before and after Treatment

The study found that the levels of CD3+, CD4+, and CD4+/CD8+ in the serum of the two groups of patients after treatment were significantly increased while the level of CD8+ was significantly decreased (*P* < 0.05), and the changes of the above indicators in the observation group were more obvious than those in the control group (*P* < 0.05), as shown in Table 4.

### 3.4. Changes of HIF1*α* and VEGF Levels in the Two Groups of Patients before and after Treatment

The study found that the serum levels of CHIF1*α* and VEGF in the two groups of patients were significantly decreased after treatment (*P* < 0.05), and the changes of the above indicators in the observation group were more obvious than those in the control group (*P* < 0.05), as shown in Table 5.

## 4. Discussion

Liver cancer has become one of the most common malignant tumors that threaten human health and survival. At present, the clinical treatment is mainly based on the clinical stage of the patient's tumor. Patients with liver cancer in the early stage can be treated with surgery, and the clinical effect and prognosis of the patients are better. Patients with tumors in the middle and advanced stages who are not suitable for surgery can be treated with hepatic arterial chemoembolization. In radiofrequency ablation, electrodes are placed in the tumor tissue and then high-frequency radio waves are emitted. In this study, when analyzing the effect of hepatic arterial chemoembolization combined with radiofrequency ablation on liver function and immune function in patients with liver cancer, it was found that the total effective rate of the observation group was significantly higher than that of the control group. The results of the study showed that after treatment, the levels of serum transaminases ALT, AST, CD8+, HIF1*α*, and VEGF were significantly decreased, and the levels of total bilirubin, direct bilirubin, indirect bilirubin, CD3+, CD4+, and CD4+/CD8+ were significantly increased, suggesting that liver arterial chemoembolization combined with radiofrequency ablation has a significant effect on liver function and immune function in patients with liver cancer, which may be related to its abnormal effect on HIF1*α* and VEGF levels.

Existing studies have shown that compared with transcatheter hepatic artery embolization, hepatic arterial chemoembolization is more effective and safe for interventional therapy of primary liver cancer [8], and hepatic arterial chemoembolization combined with radiofrequency ablation is used for primary liver cancer. Patients with liver cancer can improve clinical efficacy, reduce tumor diameter, and have a lower incidence of adverse reactions [9]. Gemcitabine combined with cisplatin has obvious effect on the treatment of liver cancer patients through TACE, without increasing the toxic and side effects, and for the non-surgical resection of hepatocellular carcinoma, the short-term efficacy of percutaneous thermal ablation is better than that of TACE [10, 11]. At the same time, RFA combined with TACE has good short-term and long-term efficacy in the treatment of primary liver cancer [12]. This study also found that the total effective rate of the observation group was significantly higher than that of the control group, and the serum transaminase ALT, AST, and CD8+ levels were significantly decreased after treatment. The levels of total bilirubin, direct bilirubin, indirect bilirubin, CD3+, CD4+, and CD4+/CD8+ were significantly increased, suggesting that hepatic arterial chemoembolization combined with radiofrequency ablation can significantly improve liver function and immune function in patients with liver cancer of recovery. However, previous studies have not analyzed the expression of cell proliferation and microenvironment hypoxia-related molecules before and after treatment in patients. The rapid proliferation of malignant tumor cells is usually accompanied by hypoxia in the microenvironment, and the rapid angiogenesis process also requires enhanced expression of vascular endothelial growth factor [13, 14]. TRAP1 is highly expressed in HepG2 cells, and it may be one of the pathways by which HIF-1*α* regulates the EMT of HepG2 hepatoma cells. There is a significant correlation between the common syndromes of primary liver cancer and serum AFP and VEGF [15, 16]. Knockdown of HIF-1 and AKT expression can inhibit the proliferation of human liver cancer cell line SMMC-7721. HIF-1 may be the main determinant of liver cancer cell proliferation. Downregulation of HIF-1 expression level can inhibit the proliferation of liver cancer cells, and knockdown of AKT expression can inhibit the proliferation of liver cancer cells, reduce the expression level of HIF-1, and synergize with the low expression of HIF-1 to inhibit the proliferation of liver cancer cells [17], and metuximab combined with TACE sequential surgery in the treatment of primary liver cancer can inhibit the high expression of VEGF and AFP, improve survival rate, reduce the rate of metastasis and recurrence, and improve the quality of life [18]. Hypoxia can induce HIF-1 in liver cancer tissue ɑ expression and immunosuppression, silencing HIF-1 β. It can inhibit the growth of transplanted tumor and provide new ideas for reversing the immunosuppression of liver cancer [19]. The high expression of HIF-1a and VEGF in the microenvironment of primary liver cancer tissue is closely related to angiogenesis, and they may be the key factors in promoting the formation of new blood vessels in the intratumoral environment and the inflammatory response in the extratumoral environment [20], and *Lycium barbarum* polysaccharide can inhibit the migration and invasion of liver cancer cells, and its mechanism may be related to the direct inhibition of VEGF [21]. This study also found that the levels of HIF1*α* and VEGF in serum of the two groups of patients were significantly decreased after treatment, suggesting that hepatic arterial chemoembolization combined with radiofrequency ablation has a significant effect on liver function and immune function in patients with liver cancer and may affect the abnormal levels of HIF1*α* and VEGF. In future research, we will further use immunohistochemistry to analyze the expression and localization of related proteins and use animal models to analyze the dynamic changes of related protein expression during the treatment process, so as to pass the reference for more reasonable clinical treatment.

Therefore, hepatic arterial chemoembolization combined with radiofrequency ablation has obvious effect on liver function and immune function in patients with liver cancer, which may be related to the regulation of abnormally expressed HIF1*α* and VEGF levels in vivo.

## Figures and Tables

**Table 1:** Comparative analysis of the clinical effective rate of treatment in the two groups of patients.

Group	Number of cases	CR	PR	SD	*P*D	Total efficiency (%)
Control group	85	10	35	27	13	72 (84.7)
Test group	85	19	50	11	5	80 (94.1)
*x* ^2^						3.977
*P*						0.046

**Table 2:** Changes of transaminase levels before and after treatment in two groups of patients.

Group	Number of cases	AST (U/L)			ALT (U/L)		
		Before treatment	After treatment	*t*/*P*	Before treatment	After treatment	*t*/*P*
Control group	85	98.6 ± 11.3	57.8 ± 7.32	3.102/0.002	90.8 ± 8.54	54.6 ± 8.32	2.745/0.008
Test group	85	99.5 ± 10.4	45.5 ± 8.33	2.915/0.004	92.6 ± 9.91	41.7 ± 7.88	2.718/0.001
*t*		0.540	10.226		1.269	10.379	
*P*		0.589	<0.001		0.206	<0.001	

**Table 3:** Changes of bilirubin levels before and after treatment in two groups of patients.

Group	Total bilirubin (*μ*mol/L)			Direct bilirubin (*μ*mol/L)			Indirect bilirubin (*μ*mol/L)		
	Before treatment	After treatment	*t*/*P*	Before treatment	After treatment	*t*/*P*	Before treatment	After treatment	*t*/*P*
Control group	23.5 ± 2.84	35.4 ± 4.88	4.735/0.002	6.22 ± 1.01	9.89 ± 1.13	3.612/0.004	15.7 ± 2.54	22.5 ± 3.91	5.975/0.000
Test group	23.7 ± 3.09	42.4 ± 3.12	3.498/0.003	6.14 ± 0.94	12.6 ± 2.98	5.876/0.000	15.4 ± 2.12	27.7 ± 3.09	4.633/0.001
*t*	0.439	11.142		0.535	7.839		0.836	9.619	
*P*	0.661	<0.001		0.594	<0.001		0.404	<0.001	

**Table 4:** Comparison of changes in immune function indexes of two groups of subjects.

Group		CD3+	CD4+	CD8+	CD4+/CD8+
Control group	Before treatment	42.5 ± 6.54	30.8 ± 4.32	18.5 ± 2.99	1.66 ± 0.49
	After treatment	55.6 ± 7.98	36.8 ± 3.99	14.3 ± 3.52	2.27 ± 0.65
*t*		11.706	9.407	8.384	6.909
*P*		0.000	0.000	0.000	0.000
Test group	Before treatment	43.6 ± 8.43	31.9 ± 4.32	19.2 ± 3.61	1.66 ± 0.57
	After treatment	59.6 ± 9.21^a^	42.7 ± 5.38^a^	11.6 ± 2.99^a^	3.68 ± 0.78^a^
*t*		11.815	14.431	14.948	19.278
*P*		<0.001	<0.001	<0.001	<0.001

*Note.* Compared with the control group, ^a^*P* < 0.05.

**Table 5:** Changes of HIF1*α* and VEGF levels before and after treatment in the two groups of patients.

Group	Number of cases	HIF1*α* (*μ*g/L)			VEGF (*μ*g/L)		
		Before treatment	After treatment	*t*/*P*	Before treatment	After treatment	*t*/*P*
Control group	85	23.6 ± 4.32	17.5 ± 4.88	6.398/0.004	40.4 ± 7.98	33.6 ± 5.88	5.284/0.009
Test group	85	24.7 ± 5.07	13.7 ± 2.98	5.365/0.005	40.9 ± 6.82	26.9 ± 5.22	4.968/0.008
*t*		1.523	6.127		0.439	7.856	
*P*		0.129	<0.001		0.661	<0.001	

## Data Availability

The data can be obtained from the corresponding author upon reasonable request.
